The article "Multi-Slice Spiral Computed Tomography Image Features under Hybrid Iterative Reconstruction Algorithm in Staging Diagnosis of Bladder Cancer" was retracted in 2023. Reasons: signs of a paper mill; suspected computer-generated content; unreliable results or conclusions; concerns about the data.

# Multi-Slice Spiral Computed Tomography Image Features under Hybrid Iterative Reconstruction Algorithm in Staging Diagnosis of Bladder Cancer

**DOI:** 10.1155/2021/7733654

**Published:** 2021-10-27

**Authors:** Lan Zang

**Affiliations:** Department of Radiology, Hangzhou Future Sci-tech City Hospital, Hangzhou 311100, Zhejiang, China

## Abstract

**Objective:**

This study was aimed to explore the accuracy of multi-slice spiral computed tomography (CT) scan in preoperative staging diagnosis of bladder cancer based on hybrid iterative reconstruction algorithm, so as to provide a more reasonable supporting basis for guiding clinical work in the future.

**Methods:**

Retrospectively, 120 patients admitted to hospital from July 2019 to April 2021, who were confirmed to be with urothelial carcinoma of the bladder by pathological examination after surgical treatment, were selected. CT images before processing were set as the control group and those after processing were set as the observation group according to whether they were processed by the hybrid iterative algorithm. Postoperative pathological examination was utilized as the standard for analysis. The accuracy and consistency of the two methods were compared.

**Results:**

The accuracy of the results of each stage of the observation group (T1 stage: 91.09%, T2 stage: 89.66%, T3 stage: 88.89%, and T4 stage: 88.89%) and consistency (T1 stage: 0.66, T2 stage: 0.69, T3 stage: 0.71, and T4 stage: 0.82) were higher than those of the control group (accuracy: T1—57.01%, T2—48.28%, T3—44.44%, and T4—44.44%). The consistency was as follows: T1—0.32, T2—0.24, T3—0.37, and T4—0.43, and the comparison was statistically significant (*P* < 0.05).

**Conclusion:**

The adoption value of the image features based on the hybrid iterative reconstruction algorithm in the diagnosis of bladder cancer staging was higher than that of the conventional multi-slice spiral CT, indicating that the hybrid iterative reconstruction algorithm had a good adoption prospect in clinical examination.

## 1. Introduction

Bladder cancer is a malignant tumor originating from urinary mucosal epithelial cells and is also one of the most common urinary malignancies, with its incidence ranking first among all genitourinary tumors in China [1–3]. There is no limit to the age of onset of the disease, which can even occur in children, and the incidence of the disease will increase with the increase of age, with a high incidence between 50 and 70 years old [4, 5]. According to statistical reports, the incidence of bladder cancer in males is 3–4 times that of females [6]. Bladder cancer is also characterized by multiple, high recurrence rate, high malignancy, low survival rate, and rapid progression [7]. Therefore, the treatment of bladder cancer has become the focus of attention, and the choice of treatment depends on the clinical staging of bladder cancer. According to statistics, the misdiagnosis rate of clinical staging of bladder cancer is about 25%–50% [8]. At present, the commonly utilized detection methods of bladder cancer in clinical mainly include B-mode ultrasound, computed tomography (CT), magnetic resonance imaging (MRI), and cystoscopy. However, B-mode ultrasound, MRI, and cystoscopy all have various limitations. For example, the resolution of the B-mode ultrasound is low, and the cystoscope will cause damage to the patient. CT is insufficient in the detection of small lesions, with staging accuracy of about 64%–92% [9–11], and CT examination has high radiation. Compared with conventional CT, helical enhanced CT can better display the size, number, and lesions of the tumor, as well as the infiltration of the tumor to some extent. However, the overall accuracy of CT in predicting tumor staging is only 60% in routine clinical examination [12], which makes people question its clinical staging.

With the rapid development of science and technology, the optimization of image algorithms is becoming more and more important [13, 14]. CT image reconstruction algorithm is the most important algorithm in the whole imaging image chain. At present, the most utilized image reconstruction algorithm is filtered back projection (FBP). Although this algorithm has the advantages of short reconstruction time and fast speed, image noise will be introduced at the same time to obscure the details of the image and indirectly increase the radiation dose [15]. Therefore, some people put forward an iterative reconstruction algorithm, which can greatly reduce the image noise, indirectly improve the image quality, and reduce the radiation dose, which has great clinical adoption value [16].

Therefore, in this study, multi-slice spiral CT images based on mixed iterative reconstruction denoising algorithm were used to detect and diagnose bladder cancer patients. The diagnostic results were compared with postoperative pathological diagnosis results to evaluate the accuracy of multi-slice spiral CT scan based on mixed iterative reconstruction algorithm in preoperative staging diagnosis of bladder cancer. It was hoped to provide a more reasonable auxiliary research basis for CT scanning technology in guiding clinical work.

## 2. Methods

### 2.1. Multi-Slice Spiral CT Based on Hybrid Iterative Reconstruction Algorithm

#### 2.1.1. The Basic Idea of Hybrid Iterative Reconstruction

The hybrid iterative algorithm first performs an initial FBP algorithm using weights and then uses two different correction loops. The first is the recursive iteration of the original data space, eliminating the noise in the raw data field and adding more steps to verify the original data. The detected deviation is utilized in the weighted FBP to generate an updated image (Figure 1).

#### 2.1.2. The Specific Process of Hybrid Iterative Reconstruction

The hybrid iterative algorithm is mainly based on noise reduction in the front and rear projection domain. Studies found that the projection data received by the CT detector approximately conform to the Gaussian distribution. The mean and variance of the projection data after logarithmic transformation conform to the following expressions:

(1) $$\begin{array}{c} \alpha_{i}^{2}=f_{i}*\;\exp\frac{q_{i}}{℘}. \end{array}$$

In equation (1), the mean value of the data received by the *i*-th detector unit is *q*_*i*_, and the variance of the data is *α*_*i*_^2^. The iteration coefficient is represented by *℘*. *f* is the target image. After that, the weighted least squares method weighted least squares (WLS) [17] is utilized to reduce the image noise in the front and rear projection space. The iterative expression of the front and back projection domain is as follows.

Front projection domain iteration is expressed as follows:

(2) $$\begin{array}{c} ℑ\left(q\right)={\left(\bar{y}-q\right)}^{\prime }\sum^{-1}\left(\bar{y}-q\right). \end{array}$$

Postprojection domain iteration is expressed as follows:

(3) $$\begin{array}{c} ℑ\left(w\right)={\left(\bar{y}-Ew\right)}^{\prime }\sum^{-1}\left(\bar{y}-Ew\right), \end{array}$$

where *q* = *Ew* is the vector of the complete projection dataset, *w* is the attenuation coefficient that needs to be calculated eventually, *E* is the projection matrix, and *y* is the logarithmic result of the detector measurement data.

Penalized weighted least squares (PWLS) algorithm [18] is introduced to improve the checkerboard effect of the traditional least squares method and ensure the convergence performance. The expression is as follows:

(4) $$\begin{array}{c} ℜ\left(E\right)={\left(\bar{T}-E\right)}^{\prime }\sum^{-1}\left(\bar{T}-E\right)+\beta R\left(e\right), \end{array}$$

where *E* is the ideal value of the estimated projection data, ∑^−1^ is the noise variance matrix, $\bar{T}$ represents the actual measured projection data, *R*(*e*) is the marked penalty factor, and *β* is the coefficient for adjusting the degree of calculation.

The guide value of each pixel on the CT image is set as *j*, then the pixel value at the center of the image is *N*_*j*_, the value of adjacent pixels is *E*_*n*_, and the weight is *U*_*jk*_. The expression of the iterative equation is as follows:

(5) $$\begin{array}{c} e_{j}^{l+1}=\frac{E_{j}+\beta \alpha_{j}^{2}\left(\sum_{k\in N_{j}^{2}}U_{jn}p_{n}^{l+1}+\sum_{k\in N_{j}^{2}}U_{jn}p_{n}^{l}\right)}{1+\beta \alpha_{j}^{2}\sum_{k\in N_{j}^{2}}U_{jn}}, \end{array}$$

where *l* is the iteration period and *N* and *E* are the adjacent regions around the target pixel.

The relationship between the preprocessed and estimated projection data is as follows:

(6) $$\begin{array}{c} R\left(e\right)=\frac{1}{2}{\sum_{j}\sum_{MeN_{j}}U_{jk}\left(E_{j}-E_{n}\right)}^{2},\\ e=\arg\underset{e\geq 0}{\min}ℜ\left(e\right). \end{array}$$

According to the analysis of the previous equation, the specific calculation steps for the iteration of the front and back projection domain are as follows.

The original projection data are calculated with the following equations:

(7) X¯=FBPy¯,q=EX¯,∑=di  agαi2qi=di  agfiexpqi℘,r¯=y¯−q,Tj=Ej′∑−1E,j∀j,αj=Tj+β′∑k∈NjUjk.

The individual pixel iterations are processed as follows:

(8) $$\begin{array}{c} {\bar{U}}_{j}^{l}≔{}_{\bar{U}}^{j},\\ {\bar{W}}_{j}^{l+1}≔\frac{E_{j}^{\prime }\sum {}^{-1}\bar{r}+T_{j}{\bar{W}}_{j}^{l}+\beta \sum_{k\in N_{j}}U_{jk}{\bar{W}}_{k}}{\alpha_{j}},\\ {\bar{W}}_{j}≔\max\left\{0,\left(1-u\right){\bar{W}}_{j}^{l}+u{\bar{W}}_{j}^{l+1}\right\},\\ \bar{r}≔\bar{r}+e_{j}\left({\bar{W}}_{j}^{l}-{\bar{W}}_{j}\right),\\ {\bar{\alpha }}_{i}^{2}≔f_{i}\exp\left(\sum_{j}E_{ij}\frac{W_{j}}{℘}\right), \end{array}$$

where *k* is the number of iteration loops and *P*_*ij*_ represents the unit data in the projection data. During the iteration process, the precalculated weight coefficient is a fixed value. The end of the iteration loop depends on the convergence requirements.

### 2.2. Research Objects

In this study, patients admitted to the hospital from July 2019 to January 2021 were retrospectively selected, who were confirmed to be with urothelial carcinoma of the bladder by pathological examination after surgical treatment. A total of 120 patients with preoperative staging using multi-slice enhanced spiral CT were included in the study. There were 93 males and 27 females, aged 42–84 years (mean age 64 ± 5.2 years). According to whether the multi-slice enhanced spiral CT images of patients with bladder cancer were processed by the hybrid iterative algorithm, the preprocessed CT images were set as the control group, and the postprocessed CT images were set as the observation group. The results of the two groups of CT images were analyzed according to the standard of postoperative pathological examination. This study had been approved by the Medical Ethics Committee, and all patients had signed the informed consent form.

Inclusion criteria were as follows: all patients had undergone surgery; no patients had distant metastases; and the patients were staged by multi-slice spiral CT before surgery, and the staging basis is shown in Table 1.

Exclusion criteria were as follows: CT imaging with severe artifacts, dislocation, noise, and calcified plaques; patients with severe liver and kidney insufficiency, heart failure, and other severe insufficiency; and patients with a history of urinary system diseases.

### 2.3. Examinations

All patients were examined by the same 64-slice spiral CT scanner, and the specific procedures were as follows.

Preparation before scanning is done as follows: patients were fasted for 8 hours and filled in the bladder (drink 1000–1500mL of water 1.5–2h before the CT scanning).  Figure 2 shows the detailed scanning process. CT images of all patients were collated and processed using a hybrid iterative reconstruction algorithm. All patients were examined by the same highly qualified and experienced physician, and radiographs were reviewed by two physicians simultaneously.

### 2.4. Observation Indexes

- The pathological examination results of patients were collected during and after operation, including the location, diameter, base, and number of bladder cancer lesions and the staging results of postoperative histopathological examination. The TNM staging method, 7th edition 2009, International Union Against Cancer was utilized for the pathological staging of bladder cancer, as presented in Table 2.
- The review results of CT images of the two groups were collated and observed, including the size, number, and location of bladder cancer lesions, the involvement of organs near bladder, and pelvic lymph node metastasis. The preoperative CT staging of bladder cancer was obtained.
- Comparison of multi-slice spiral CT staging and pathological staging of bladder cancer was implemented between the two groups. The number of tumors in each stage was statistically analyzed, and the accuracy of staging diagnosis of the two groups of CT images was analyzed.

### 2.5. Statistical Analysis

The SPSS 22.0 statistical system was utilized for data entry, sorting, and statistical analysis. The comparison of count data was performed by *χ*^2^ test, and the comparison of measurement data was performed by *t*-test. In addition, the comparison of the mean of multiple samples adopted the analysis of variance, the lysergic acid diethylamide (LSD) method was utilized when the variance was uniform, and the Dunnett T3 method was utilized when the variance was uneven. The kappa test was performed on the consistency between the results of the two groups of multi-slice spiral CT examination and the comprehensive diagnosis. When kappa>0.75, the consistency between the two was strong. When 0.4≤kappa<0.75, the consistency between the two was general. When kappa <0.4, the consistency between the two was poor. *P* < 0.05 was statistically different.

## 3. Results

### 3.1. Verification Results of the Hybrid Iterative Reconstruction Algorithm

The 120 kV/200 mA FBP algorithm and the 120 kV/90 mA hybrid iterative reconstruction algorithm were utilized for clinical verification. The effects of different parts are shown in Figure 3 (abdomen), Figure 4 (brain), and Figure 5 (chest). The results all showed that under the condition of reducing the radiation dose, the hybrid iterative reconstruction algorithm maintained the image quality, met the needs of clinical diagnosis of different visceral diseases, and can be utilized in this experimental study.

### 3.2. Comparison of General Patient Information

Of the 120 cases of bladder cancer studied, 93 were males and 27 were females, with a male-to-female ratio of 3.44 : 1 and an age range of 42–84 years (average age of (64 ± 5.2) years). There were 82 cases with single lesions and 33 cases with multiple lesions (31.2%). The total number of cancer foci was 163. Among the 120 patients, most of them were male, and the elderly were the main group of patients with the peak incidence between 60 and 80 years old. 81.13% of the patients were over 60 years old.  Figure 6 shows the specific distribution.

### 3.3. Statistics of Pathological Examination Results

According to the statistical results of intraoperative and postoperative pathological examination, the following results were obtained. Tumor diameter of 163 bladder cancer lesions ranged from 0.5 cm to 7.7 cm.  Figure 7 shows the specific distribution. The basal condition of the tumor lesions was divided into three categories. According to the classification, there were 82 with pedicle, 75 with wide base, and 3 with unrecognizable basal condition. For tumor sites, 84 tumors occurred in the middle wall, 39 tumors occurred in the posterior wall, 19 tumors occurred in the trigonometric region of the bladder, 17 tumors occurred in the parietal wall, and 4 tumors occurred in the anterior wall. The surgical pathological stages showed that there were 107 cases at T1 stage, 29 cases at T2 stage, 18 cases at T3 stage, and 9 cases at T4 stage, and the proportions are shown in Figure 8.

### 3.4. Comparison of the Results of CT Image Examination and Pathological Examination between the Two Groups

Through statistical analysis, the following results were obtained. In terms of the number of cancer lesions, the CT results of the two groups were consistent with the pathological results, both suggesting 163 lesions, and the difference was not considerable (*P* > 0.05). In terms of lesion diameter, the distribution of the three groups of data is shown in Figure 9. After analysis and comparison, it was found that the diameter distribution of the observation group was closer to the pathological examination results. The distribution in different diameters was 0.5–0.9 cm for 12 lesions, 1.0–1.9 cm for 49 lesions, 2.0–2.9 cm for 48 lesions, 3.0–3.9 cm for 24 lesions, and ≥4.0 cm for 29 lesions. There was no considerable difference in the distribution (*P* > 0.05). In terms of tumor sites, the 160 tumors found in the observation group were as follows. There were 84 in the middle wall, 38 in the posterior wall, 18 in the trigonometric region of the bladder, 17 in the parietal wall, and 3 in the anterior wall. In the control group, the results showed that there were 83 in the middle wall, 37 in the posterior wall, 18 in the trigonometric region of the bladder, 17 in the parietal wall, and 3 in the anterior wall. There was no considerable difference in the distribution of 158 specimens (*P* > 0.05). In terms of tumor staging results, the CT staging results of the two groups were as follows. In the observation group, 95 tumors were at T1 stage, 36 tumors were at T2 stage, 23 tumors were at T3 stage, and 9 tumors were at T4 stage. In the control group, 71 were at T1 stage, 50 were at T2 stage, 30 were at T3 stage, and 12 were at T4 stage. Comparison of pathological stages is shown in Table 3.

### 3.5. Comparison of the Accuracy and Consistency of the Two Groups of CT Image Staging Results

According to the calculation and analysis in Table 3, taking the pathological staging results as the standard, the accuracy of CT image staging results in the observation group was 91.09% for T1, 89.66% for T2, 88.89% for T3, and 88.89% for T4. The consistency was 0.66 for T1, 0.69 for T2, 0.71 for T3, and 0.82 for T4. The accuracy of the control group was 57.01% for T1, 48.28% for T2, 44.44% for T3, and 44.44% for T4. The consistency was 0.32 for T1, 0.24 for T2, 0.37 for T3, and 0.43 for T4. After analysis and comparison, it was found that the accuracy and consistency of the results of each stage in the observation group were higher than those in the control group, and the comparison was considerable (*P* < 0.05), as illustrated in Figures 10 and 11.

## 4. Discussion

Clinical statistical analysis showed that the main group of bladder cancer is the elderly, and the incidence rate of males is much higher than that of females. The most common sites are the lateral and posterior walls of the bladder [19–21]. According to the statistics of this study, among the 120 cases of bladder cancer, the ratio of male to female was 3.44 : 1, and the incidence peak was between 60 and 80 years old. 81.13% of the cases were patients over 60 years old. Among the 163 tumors, 84 tumors occurred in the lateral wall, 39 tumors occurred in the posterior wall, and 40 tumors occurred in other parts. The results were consistent with the above statistical results. Then, the CT images of the observation group and the control group were compared with the pathological diagnosis results in terms of the number of cancerous lesions, the diameter of lesions, and the diagnosis of tumor sites, and the results showed no considerable differences. It was suggested that the processing effect of the hybrid iterative reconstruction algorithm was not reflected in the above aspects. However, the value of the technique has been demonstrated in terms of pathological staging. The results showed that the accuracy and consistency of each stage of diagnosis in the observation group were higher than those in the control group. The accuracy of each period was above 88%, while the kappa value was above 0.65, which fully reflected the value of the hybrid iterative reconstruction algorithm in the staging diagnosis of bladder cancer. Löve et al. [22] conducted a study using a hybrid iterative reconstruction algorithm to improve the image quality of craniocervical CT angiography. Results showed that iterative reconstruction algorithm significantly improved the image quality of craniocervical CT, especially at the thoracic inlet. A study on the effect of high pitch protocol and hybrid iterative reconstruction algorithm on the image quality of brain subtraction 3D CT angiography showed that 3D-CTA with high pitch protocol and HIR can reduce radiation dose while reducing venous enhancement and image noise to an adequate diagnostic level [23]. The above studies all supported the adoption value of the hybrid iterative reconstruction algorithm. However, the staging results of this study indirectly illustrated the limitations of multi-slice spiral CT in the preoperative staging of bladder cancer. Some experts applied multi-slice spiral CT and MRI in the diagnosis of prostate cancer at different stages to analyze the application value of the two methods. The results showed that both MRI and MSCT can accurately detect stage C and stage D of prostate cancer. The ADC value in MRI is of great clinical significance in determining the risk of tumor. The conclusion was that MRI was more valuable than MSCT in the diagnosis of prostate cancer at different stages [24]. There were two methods utilized to diagnose peritoneal metastases from primary ovarian cancer, and the results also indicated that MRI was more accurate in the diagnosis of peritoneal metastasis in ovarian cancer patients compared with multi-slice spiral CT [25]. However, it was not universal and may be more effective than other screening methods. A study comparing the value of IVP and multi-slice spiral CT in the diagnosis of bladder cancer showed that compared with IVP, multi-slice spiral CT had a significantly higher detection rate of bladder cancer with better scanning and diagnostic positioning. It can more clearly display the tissue structure of bladder cancer lesions, which was more conducive to providing a strong diagnostic basis [26].

## 5. Conclusion

In conclusion, the image features of multi-slice spiral CT based on the hybrid iterative reconstruction algorithm had higher adoption value in the diagnosis of bladder cancer staging than the conventional multi-slice spiral CT, indicating that the hybrid iterative reconstruction algorithm had a good adoption prospect in clinical examination. However, the case data of this study are limited, and the sample size is small, which lacks the representativeness of large samples. We will make further improvements in future studies. However, from this study, it was found that deep learning algorithms had good development prospects in the auxiliary diagnosis of medical imaging.

## Figures and Tables

**Figure 1:** Algorithm principle of hybrid iteration.

**Figure 2:** Scanning process and parameters.

**Figure 3:** Comparison of abdominal images under FBP algorithm and hybrid iterative algorithm. (a) FBP. (b) Mixed iteration.

**Figure 4:** Comparison of brain images under FBP algorithm and hybrid iterative algorithm. (a) FBP. (b) Mixed iteration.

**Figure 5:** Comparison of chest images under FBP algorithm and hybrid iterative algorithm. (a) FBP. (b) Mixed iteration.

**Figure 6:** Age distribution.

**Figure 7:** Diameter distribution.

**Figure 8:** Pathological stages.

**Figure 9:** Diameter distribution of the three sets of results.

**Figure 10:** Comparison of the accuracy of the staging results of the two groups. ^∗^indicated that the comparison is statistically significant, *P* < 0.05.

**Figure 11:** Comparison of the consistency of the staging results of the two groups. ^∗^indicated that the comparison is statistically significant, *P* < 0.05.

**Table 1:** CT staging of bladder cancer.

Stages		Imaging features
T1		Lump in the bladder cavity and smooth bladder wall without thickening.
T2	T2a	The bladder wall was thickened, but there was no local stiffness.
	T2b	The bladder wall was thickened and stiff, but the outer margin was smooth.
T3		Bladder wall was thickened and irregular, with blurred boundaries, and there was soft tissue density shadow in the surrounding fat layer.
T4		Tumor invaded adjacent organs. When the tumor invaded the seminal vesicle, the angle of the bladder seminal vesicle disappeared. When the tumor invaded the prostate, the boundary of the prostate was not clear and the density was uneven.

**Table 2:** Pathological staging of bladder cancer using the 7th edition of TNM staging method, 2009.

T (primary tumor)	Tx		The primary tumor could not be evaluated.
	To		No evidence of primary tumor.
	Ta		Non-invasive papillary carcinoma.
	Tis		Carcinoma in situ (“squamous carcinoma”).
	T1		Tumor invasion of subepithelial connective tissue.
	T2 (muscular layer invasion)	T2a	Tumor invasion of superficial muscularis (medial half).
		T2b	Tumor invasion of the deep muscle layer (lateral half).
	T3 (surrounding tissue invasion)	T3a	The tumor invaded the tissues around the bladder under the microscope.
		T3b	The tumor can be seen to invade the tissues around the bladder (extra-bladder mass).
	T4 (other organ or tissue invasion)	T4a	The tumor invaded the prostate, uterus, or vagina.
		T4b	Tumor invaded the pelvic or abdominal wall.

N (regional lymph nodes)	Nx		Regional lymph nodes could not be evaluated.
	No		No regional lymph node metastasis.
	N1		Single lymph node metastasis from the true pelvic region (internal iliac, obturator, external iliac, or anterior sacral).
	N2		Multiple lymph nodes in the true pelvis (internal iliac, obturator foramen, external iliac, or anterior sacral).
	N3		Common iliac lymph node metastasis.

M (distant metastasis)	Mx		Distant metastases could not be assessed.
	M0		No distant metastasis.
	M1		There were distant metastases.

**Table 3:** The staging results of different groups.

Group		Pathological staging (pieces)				Total (pieces)
		T1	T2	T3	T4	
Observation group (cases)	T1	92	3	0	0	95
	T2	9	26	1	0	36
	T3	6	0	16	1	23
	T4	0	0	1	8	9
Total (cases)		107	29	18	9	163

Control group (cases)	T1	61	10	1	0	71
	T2	36	14	1	1	50
	T3	12	5	8	4	30
	T4	0	0	8	4	12
Total (cases)		107	29	18	9	164

## Data Availability

The data used to support the findings of this study are available from the corresponding author upon request.
